# Clinical Characteristics and Risk Factors for Pulmonary Infection in Emergency ICU Patients

This article has been retracted.

**DOI:** 10.1155/2022/7711724

**Published:** 2022-04-29

**Authors:** Yan Zhang, Hui Cao, Xiang Gong, Yang Wu, Peng Gu, Linling Kong, Limeng Wu, Jiali Xing

**Affiliations:** ^1^Department of Infection, Nantong First People's Hospital, No. 6, Haier Lane North Road, Nantong, Jiangsu 226000, China; ^2^Department of Rehabilitation, Nantong First People's Hospital, No. 6, Haier Lane North Road, Nantong, Jiangsu 226000, China; ^3^Department of Emergency, Nantong First People's Hospital, No. 6, Haier Lane North Road, Nantong, Jiangsu 226000, China

## Abstract

**Background:**

Pulmonary infection in the emergency ICUs increases patient morbidity, hospital stay, treatment costs, and the risk of related adverse events.

**Methods:**

This study included 695 patients admitted to our emergency ICU between December 2019 and March 2021. Medical records of emergency ICU patients were reviewed to collect their clinical data, including antibiotic use, history of tracheostomy, history of mechanical ventilation, presence or absence of underlying disease, history of smoking, alcohol consumption, age, gender, and history of shock. Bacterial cultures were performed. The incidence, main clinical features, main pathogens, and risk factors of pulmonary infection in emergency ICU were analyzed.

**Results:**

In this study, 69 of the 695 emergency ICU patients (9.93%) developed pulmonary infection. The main clinical features of patients with pulmonary infection included cough and expectoration (97.10%), shortness of breath and chest tightness (95.65%), leukocyte elevation (69.57%), confusion (31.88%), drowsiness (28.99%), persistent fever (27.54%), and nausea and vomiting (10.14%). The main pathogenic bacteria in those with pulmonary infection included *Klebsiella pneumoniae* (62.32%), *Pseudomonas aeruginosa* (49.28%), *Streptococcus pneumoniae* (21.74%), *Staphylococcus aureus* (39.13%), *Candida albicans* (7.25%), *Pneumococcus pneumoniae* (15.95%), *Pseudomonas aeruginosa* (24.64%), and lung diplococcus inflammatory (13.04%). Univariate analysis showed that there were no significant differences in the occurrence of pulmonary infection with regard to sex, smoking, and alcohol consumption, but there were significant differences with regard to age, basic disease, invasive surgery, and shock. Logistic regression analysis confirmed that age ≥ 80 years, invasive surgery, shock, and basic diseases ≥ 2 were important risk factors for pulmonary infection in emergency ICU patients.

**Conclusion:**

Considering the clinical features and risk factors for pulmonary infection in the emergency ICU, preventive and control measures are required to minimize its occurrence and ensure good outcomes.

## 1. Introduction

Pulmonary infection is caused by inhalation injury, tracheostomy or intubation, suppurative thrombophlebitis, invasive wound infection, atelectasis, surgical anesthesia, pulmonary edema, shock, and aspiration [1, 2], and patients often have different degrees of increased sputum volume, fever, and cough, among other manifestations [3–5].

Patients in the intensive care unit (ICU), especially gerontal patients, are critically ill and frequently have multiple diseases due to poor resistance, decreased body immunity, and obvious degradation of body function, and they have a higher incidence of pulmonary infection [6]. Pulmonary infections are particularly severe in emergency ICU patients, leading to increased risk of patient morbidity, length of hospital stay, treatment costs, and associated adverse events, which can negatively impact disease outcomes [7–9]. In addition, in recent years, with the development of rescue technology and application of new antibacterial agents, the pathogenic and clinical characteristics of pulmonary infection have also changed. Therefore, the timely identification of disease characteristics and implementation of targeted prevention and control have become the research focus [10, 11].

Therefore, this study was aimed at determining the clinical characteristics and risk factors for pulmonary infection in emergency ICU patients.

## 2. Materials and Methods

### 2.1. Patients

We selected 695 patients admitted at our emergency ICU between December 2019 and March 2021. We included (1) patients diagnosed via radiography, routine hematological tests, and comprehensive clinical tests (to assess temperature, sputum, and cough); (2) patients aged ≥18 years; (3) those with good compliance and who could cooperate during the investigation and research; and (4) individuals whose families were aware of the study and provided informed consent. The exclusion criteria were as follows: (1) patients with kidney, liver, or other organ lesion; (2) patients with a history of immunosuppressant and glucocorticoid treatment; (3) individuals with metabolic and autoimmune disease; (4) patients who died during the study period; and (5) those who voluntarily quit the study. Among 695 patients with pulmonary infection in emergency ICU, 413 were male and 282 were female; the average age was 69.46 ± 14.19 (range 46–89) years. The length of hospitalization ranged from 11 to 26 days, with an average stay of 18.91 ± 5.69 days. This study was approved by the Ethics Committee of our hospital.

### 2.2. Methods

#### 2.2.1. Baseline Data Statistics

The medical records of ICU emergency patients were reviewed by trained researchers to collect clinical data, including antibiotic use, history of tracheotomy, history of mechanical ventilation, presence or absence of underlying diseases, smoking history, drinking history, age, and gender.

#### 2.2.2. Bacterial Culture

Sputum samples were collected from all patients, inoculated in blood, phenylethanol, and MacConkey and Sabouraud medium, and cultured in a 35°C constant temperature incubator. The pathogenic bacteria and drug susceptibility were identified and analyzed by using a bioMérieux drug susceptibility tester, reagent, and bacterial identification instrument. An antibiotic susceptibility test was performed by the KB disk method and minimum inhibitory concentration method. Quality control strains included *Staphylococcus aureus* (ATCC29213), *Klebsiella pneumoniae* (ATCC700603), *Pseudomonas aeruginosa* (TCC27853), and *Escherichia coli* (ATCC25922) (provided by the Clinical Laboratory Center of National Health and Family Planning Commission).

#### 2.2.3. Indicators

The following parameters of the patients were determined as follows: the occurrence of pulmonary infection and the main clinical characteristics of patients with pulmonary infection.

#### 2.2.4. Statistical Method

SPSS version 22.0 was used for the data analysis. Continuous data are expressed as mean ± SD and were analyzed with the *t*-test. Categorical data are expressed as *n* (%) and were analyzed by the *χ*^2^ test. Multivariate logistic regression analysis was performed to identify risk factors for pulmonary infection in the emergency ICU. One-tailed *P* < 0.05 indicated statistical significance.

## 3. Results

### 3.1. Occurrence of Pulmonary Infection in Emergency ICU Patients

Sixty-nine (9.93%) out of 695 emergency ICU patients developed pulmonary infection.

### 3.2. Analysis of the Main Clinical Characteristics of Patients with Pulmonary Infection

The main clinical features of patients with pulmonary infection included cough and expectoration (97.10%), shortness of breath and chest tightness (95.65%), leukocyte elevation (69.57%), confusion (31.88%), drowsiness (28.99%), persistent fever (27.54%), and nausea and vomiting (10.14%) (Table 1).

### 3.3. Main Pathogenic Bacteria in Patients with Pulmonary Infection

The main pathogenic bacteria in those with pulmonary infection included *K. pneumoniae* (62.32%), *P. aeruginosa* (49.28%), *S. pneumoniae* (21.74%), *S. aureus* (39.13%), *C. albicans* (7.25%), *Pneumococcus pneumoniae* (15.95%), *Pseudomonas aeruginosa* (24.64%), and lung diplococcus inflammatory (13.04%) (Table 2).

### 3.4. Risk Factors for Pulmonary Infection in the Emergency ICU

From the univariate analysis, there were no significant differences in the occurrence of pulmonary infection with regard to sex, smoking, and drinking status (*P* > 0.05), but there were significant differences with regard to age, basic disease, invasive surgery, and shock (*P* < 0.05) (Table 3). Logistic regression analysis confirmed that age ≥ 80 years, invasive surgery, shock, and basic diseases ≥ 2 were important risk factors for pulmonary infection in emergency ICU patients (*P* < 0.05) (Table 4).

## 4. Discussion

Compared with those in the general ward, emergency ICU patients have more complex and serious conditions, and 90% of them have complications, leading to a poor prognosis [12–14]. Pulmonary infection is a common complication in emergency ICU patients. Recently, with the increased pressure in the medical environment and aging of the population, the problems above have worsened, and pulmonary infection can significantly increase the difficulty of disease management, which is an important preventive factor for ICU treatment failure [15–17]. Therefore, it seemed crucial to determine the clinical characteristics and risk factors for pulmonary infection in emergency ICU patients.

This study investigated the occurrence of pulmonary infection in patients in the emergency ICU of our hospital. The results showed that 9.93% of patients in the emergency ICU had pulmonary infection. Most of the patients had varying degrees of cough and sputum, shortness of breath, chest tightness, leukocyte increase, etc., and there were many bacterial causes of pulmonary infection, including *K. pneumoniae*, *P. aeruginosa*, *S. pneumoniae*, and *S. aureus*.

In order to ensure the rationality and effectiveness of treatment, clinical practice should be based on sputum culture and drug sensitivity test results for targeted drug use. This study further explored the risk factors for pulmonary infection in emergency ICU patients and found that age ≥ 80 years, invasive surgery, shock, and basic diseases ≥ 2 were important risk factors for pulmonary infection in emergency ICU patients. Possible reasons for these findings are outlined below.

In elderly patients, immune function and immune cell proliferation were significantly decreased. Therefore, the body's resistance capacity gradually weakens. In particular for the lining of respiratory mucosa and similar tissues, due to the lack of an effective protective barrier, coupled with the poor metabolic function of the elderly, the accumulation of metabolites is more obvious and the secretion increases [12].. Moreover, the movement of the mucosal cilia is weak, making it difficult to discharge secretions, which eventually leads to lung infection [18]. Therefore, for older patients in the emergency ICU, disease and vital sign assessments should be strictly performed and airway clearance should be maintained, to minimize the incidence of pulmonary infection.

Many emergency ICU patients suffer from other diseases including coronary heart disease, diabetes, and hypertension [10]. These diseases or more serious conditions can affect the blood circulation, leading to insufficient blood supply to the organs. The immune factor contained in the blood is an important factor in the body's resistance to infectious diseases. If circulation is impaired, the ability of the lungs to resist infection will be reduced. Therefore, in clinical practice, in addition to the necessary treatment for emergency ICU patients, intervention for underlying diseases should be highly emphasized to preclude their influence on the overall treatment [17].

Invasive surgery is an important factor in increasing lung infections. For ICU patients, interventions such as tracheal intubation and assisted ventilation are required during rescue [7].. In addition, invasive interventions such as the placement of an indwelling catheter, deep vein catheterization, and tracheotomy are often required. If aseptic techniques are not strictly followed during these procedures, it is easy to cause cross infection. Moreover, tracheotomy causes long-term exposure of the trachea, which increases the risk of bacterial infection [19, 20]. Therefore, it is necessary to carefully disinfect the hands and related objects during invasive surgery, as well as ensure strict adherence to aseptic techniques to prevent infection.

Shock is a disturbance of the body's microcirculation, resulting in insufficient perfusion of the lungs, brain, heart, and other organs. Abnormal lung perfusion affects the respiratory mucosal barrier function, reduces the ability of the respiratory mucosa to clear pathogenic bacteria, and increases the risk of lung infection. Therefore, for emergency ICU patients, the management of the drainage tube and tracheal intubation should be standardized, respiratory secretions should be promptly cleaned, and aseptic techniques should be carefully utilized [7].

There are some limitations of our study. Airway inflammation is a hallmark of lung infection. The study lacked an assessment of key inflammatory markers. Patients with pulmonary infection are at high risk of developing hypertension, so future studies should include basic parameters such as blood pressure and assess the correlation between hypertension and pulmonary infection. In addition, sputum culture in ICU patients to diagnose pulmonary infection flora should avoid misdiagnosis caused by common oral flora contamination.

## 5. Conclusion

In conclusion, the main clinical characteristics of patients in the emergency ICU included cough, expectoration, shortness of breath, and chest tightness, and the main pathogenic bacteria were *K. pneumoniae* and *P. aeruginosa*. Age ≥ 80 years, invasive surgery, shock, and basic diseases ≥ 2 were important risk factors for pulmonary infection in emergency ICU patients. In clinical practice, preventive and control measures can be taken to minimize the risk of pulmonary infection in the emergency ICU and ensure good patient outcomes.

## Figures and Tables

**Table 1:** Analysis of the main clinical characteristics of patients with pulmonary infection in the emergency ICU.

Clinical characteristics	Cases (*n*)	Percentage (%)
Cough and expectoration	675	97.10
Shortness of breath and chest tightness	665	95.65
Persistent fever	191	27.54
Nausea and vomiting	70	10.14
Drowsiness	201	28.99
Confusion	221	31.88
Leukocyte elevation	483	69.57

**Table 2:** The main pathogenic bacteria in patients with pulmonary infection in the emergency ICU.

Pathogenic bacteria types	Cases (*n*)	Percentage (%)
Klebsiella pneumoniae	433	62.32
Pseudomonas aeruginosa	342	49.28
Streptococcus pneumoniae	151	21.74
Staphylococcus aureus	272	39.13
Da albicans	50	7.25
Pneumococcus pneumoniae	111	15.95
Pseudomonas aeruginosa	171	24.64
Lung diplococcus inflammatory	90	13.04

**Table 3:** Univariate analysis of pulmonary infection in the emergency ICU.

Items		Cases	Infection rate	*χ* ^2^/*t* value	*P* value
Age	≥80 years old	324	48 (14.81)	15.201	0.001
	<80 years old	371	21 (5.66)		
Gender	Male	413	45 (10.90)	0.816	0.366
	Female	282	24 (8.51)		
Smoking	Yes	251	22 (8.76)	0.408	0.523
	No	444	47 (10.59)		
Drinking	Yes	302	28 (9.27)	0.257	0.612
	No	393	41 (10.43)		
Basic disease	1 species	421	27 (5.70)	13.772	0.001
	≥2 species	274	42 (15.33)		
Invasive operation	Yes	359	51 (14.21)	15.198	0.001
	No	336	18 (5.36)		
Shock	Yes	354	50 (14.12)	13.267	0.001
	No	341	19 (5.57)		

**Table 4:** Logistic regression analysis of pulmonary infection in the emergency ICU.

Variables	*β*	S.E.	Wald *χ*^2^	*P*	OR	95% CI
Age ≥ 80 years old	1.155	0.322	12.856	<0.001	3.173	1.717~5.862
Invasive operation	1.447	0.491	8.681	<0.001	4.249	2.538~7.113
Shock	1.317	0.501	6.913	<0.001	3.733	2.059~6.768
Basic disease ≥ 2 species	1.636	0.538	8.245	<0.001	5.134	3.011~8.753

## Data Availability

The authors confirm that the data supporting the findings of this study are available within the article.
